# MRI T2WI High Signal Is a Risk Factor for Perioperative Complications in Patients with Cervical Spondylosis with Spinal Cord Compression: A Propensity Matching Score Analysis

**DOI:** 10.1155/2022/8040437

**Published:** 2022-03-01

**Authors:** Shengsheng Huang, Xuhua Sun, Liyi Chen, Ming Yi, Tuo Liang, Jie Jiang, Jiarui Chen, Chong Liu, Xinli Zhan

**Affiliations:** Spine and Osteopathy Ward, The First Affiliated Hospital of Guangxi Medical University, No. 6 Shuangyong Road, Nanning, Guangxi 530021, China

## Abstract

**Objective:**

The purpose of this study was to compare the perioperative complications and clinical efficacy of patients with cervical spondylosis with spinal cord compression (CSWSCC) with or without MRI T2WIHS (T2-weighted image high signal) by means of propensity matching score grouping.

**Methods:**

We analyzed a single-center data of 913 surgical patients with CSWSCC by propensity matching score in this study, of which 326 patients had preoperative cervical MRI T2WIHS. The patient's general condition and perioperative indicators were collected. The MRI T2WIHS and normal groups were paired 1 : 1 to eliminate selection bias by propensity matching score. Finally, a total of 312 pairs were matched successfully. The results of perioperative complications and other outcome variables were compared between the two groups by Cox function analysis.

**Results:**

The postoperative blood loss, operation time, blood transfusion volume, systemic complications, local complications, volume of drainage, abnormal use of antibiotic, length of hospital stay, and JOA (Japanese Orthopaedic Association) improvement rate were analyzed. As the only complication with significant statistical difference, the incidence of IRI (ischemia-reperfusion injury) in patients with MRI T2WIHS was significantly higher. The length of hospital stay was more significantly increased in patients with MRI T2WIHS; on the contrary, the JOA improvement rate decreased significantly.

**Conclusion:**

This study confirmed that there was no significant difference in the incidence of perioperative complications in CSWSCC patients with or without MRI T2WIHS, except for the IRI. Moreover, the JOA improvement rate of patients without MRI T2WIHS was significantly better, with the length of hospital stay reduced.

## 1. Background

Long-term clinical studies have shown that the surgical treatment of CSWSCC is effective [1]. The surgical treatment of CSWSCC is mainly to relieve the compression of the spinal cord and nerves through surgical decompression so as to promote the recovery of nerve function. At present, the main surgical treatment methods include anterior cervical discectomy with or without fusion, posterior decompression with or without fusion, and anterior and posterior combined decompression with internal fixation. Magnetic resonance imaging (MRI) is very important in the diagnosis of cervical spondylosis and therapeutic significance; magnetic resonance can show clearly the case of spinal cord compression, even the pathological changes inside the spinal cord wait like edema, hemorrhage, cavity, and occupation [2, 3]. The alteration of MRI T2WI high signal (T2WIHS) is closely related to spinal cord compression and clinical severity in patients with CSWSCC [4]. At present, many studies have shown that MRI T2WIHS imaging indicates a poor prognosis of surgical treatment, and the loss of high MRI T2 imaging signal after surgery indicates a long-term good prognosis of patients [5–7]. However, to date, there have been few comparative studies on perioperative complications in patients with CSWSCC with or without MRI T2WIHS. Complications of cervical spine surgery can be very difficult for the spine surgeon, such as cerebrospinal fluid leakage (CSFL), ischemia-reperfusion injury (IRI), hoarseness, dysphagia, esophageal fistula, C5 nerve root palsy, axial pain, local hematoma, and incision infection [8–11]. In addition, it is of great significance to develop individualized countermeasures by comparing the perioperative complications of CSWSCC patients with or without MRI T2WIHS. In order to effectively eliminate the error caused by selection deviation, we used the propensity matching score analysis method in this study [12, 13].

## 2. Materials and Methods

### 2.1. Materials of the Study

In this study, we collected the clinical data of patients hospitalized for surgery in the Department of Spinal Osteopathology, the First Affiliated Hospital of Guangxi Medical University from June 2012 to June 2021 at random, and retrospectively analyzed them by propensity matching score. Of the 913 surgical patients with CSWSCC included in this study, 326 patients had preoperative cervical MRI T2 images suggesting hyperintensity. The 22 preoperative independent variables were matched 1 : 1 with the control group: gender, age, BMI (body mass index), emergency admission, FG (Frankel grading), revision surgery, OALL (ossification of anterior longitudinal ligament), OPLL (ossification of posterior longitudinal ligament), cervical instability, diabetes, hypertension, CHD (coronary heart disease), LKD (liver and kidney dysfunction), cerebrovascular disease, COPD (chronic obstructive pulmonary disease), peptic ulcer, history of malignant tumor, osteoporosis, AS (ankylosing spondylitis), RA (rheumatoid arthritis), smoking history, and surgical approach. Inclusion criteria included the following:

- Inpatients with CSWSCC from June 2012 to June 2021
- All preoperative examinations were completed
- The operation of cervical decompression and internal fixation was successfully completed

The exclusion criteria covered the following:

- Patients with nonmain diagnosis of CSWSCC after admission, such as cervical tuberculosis, cervical tumor, and cervical medullary space-occupying lesions
- Patients who have not completed cervical decompression and internal fixation
- Patients with cervical spinal cord injury due to trauma
- Patients without complete perioperative clinical and radiographic data

All patients in this research obtained informed consent, and the research was reviewed and approved by the Ethics Committee of the First Affiliated Hospital of Guangxi Medical University.

### 2.2. Result Evaluation by the Variables

Preoperative cervical spine anteroposterior and lateral, hyperextension and flexion radiographs, and cervical spine CT and MRI examinations were completed for each patient. MRI T2 images showed hyperintensity in the spinal cord in transverse, coronal, and sagittal images of the cervical spine, and the surgical segment was consistent with the segment with altered spinal signals. Preoperative and postoperative JOA (Japanese Orthopaedic Association), FG, and other scoring scales were completed, and the patient's detailed personal history was recorded. Furthermore, operating time, intraoperative bleeding, blood transfusion, dyspnea, pneumoderma, cerebrovascular accident, postoperative peptic ulcer, dysphagia, pneumonia, hoarseness, sepsis, mental disorder, DVT (deep vein thrombosis), palsy of C5, axial pain, CSFL, esophagostomy, local hematoma formation, sense of girdle, volume of drainage, incision infection, special treatment of postoperative complications, urinary tract infection, duration of perioperative antibiotic use, and hospital stay were recorded.

Moreover, other diagnostic criteria were as follows: postoperative deltoid weakness, arm pain, and arm numbness were considered as C5 root paralysis [14]. When postoperative fever, white blood cell > 10∗10^9^/L (with increased neutrophil ratio), surgical incision redness and swelling with purulent secretions, or the bacteria culture of incision secretions was positive, it was considered as incision infection [15]. Postoperative pain from the neck to around the scapula was considered axial pain [16]. Uroscopic examination of white blood cells greater than 5 per high power field, accompanied by discomfort in urination, with or without fever, was considered as urinary tract infection. CSFL was considered if the dural sac was torn during the operation, the postoperative incision drainage was clear fluid, or confirmed by MRI or ultrasound examination. Moreover, abnormal use of antibiotics was defined as more than the duration of perioperative prophylaxis for a class of incisions. After surgery, decreased neurological function or neurological impairment (decreased muscle strength and increased sensory impairment) was considered as IRI [17].

### 2.3. Statistical Analysis

The use of PSM (propensity score matching) analysis in our clinical study allowed for a good correction of selectivity bias, which was confirmed in many previous studies [18–21]. SPSS used version 22.0 (SPSS, Inc., Chicago, IL, USA), and *P* value < 0.05 was considered statistically significant. Firstly, we identified the variables of propensity matching (the MRI T2WIHS group and the normal group) as follows: gender, age, BMI, emergency admission, JOA score, FG, revision surgery, OALL, OPLL, cervical instability, diabetes, hypertension, coronary heart disease, liver and kidney dysfunction, cerebrovascular disease, COPD, peptic ulcer, history of malignant tumor, osteoporosis, AS, RA, smoking history, and surgical approach. Secondly, the *t*-test or Wilcoxon rank-sum test was used for independent samples, and the chi-square test was used for categorical variables to assess the balance of baseline characteristics between the two groups (the MRI T2WIHS group and the normal group). Four baseline characteristics, including gender, FG, cervical instability, and surgical approach, were selected as covariables of the PSM model. Moreover, the random technique, with a predefined caliper of 0.2 of the PS, with a 1 : 1 pairing, was used. Then, there was no statistical difference between the two groups of variables after matching (*d* (standardized difference) < 0.1 was considered as acceptable). Finally, Cox function was used to analyze the postoperative blood loss, operation time, blood transfusion volume, systemic complications, local complications, volume of drainage, abnormal use of antibiotic, length of hospital stay, JOA improvement rate, and other outcome variables, with multivariate regression analysis to verify.

## 3. Results

In our study, the perioperative data of 913 patients with CSWSCC were collected, as shown in Table 1. 326 patients were included in the MRI T2WIHS group, and 587 patients were included in the MRI T2 normal signal group. The proportion of males was higher in the T2WIHS group (T2WIHS/normal = 226 (69.3)/256 (43.6), *P* = 0.002) before PSM. In addition, the proportion of patients with low Frankel grading was higher in the T2WIHS group (T2WIHS/normal = 179 (54.9)/199 (33.9), *P* < 0.001), and the proportion of cervical spine instability was also significantly higher (T2WIHS/normal = 56 (17.2)/56 (9.5), *P* < 0.001) compared with the normal group. There was no significant difference in other preoperative medical history and comorbidities. After matching by propensity matching score, 312 MRI T2WIHS patients were successfully matched to 312 normal patients. The differences of preoperative case characteristics were eliminated after pairing, and all *P* values were greater than 0.05 (Table 1).

Table 2 presents the perioperative system, local complications, incision drainage, and abnormal antibiotic use in the MRI T2WIHS and general groups before and after matching. Before matching, the perioperative systemic complications of spinal cord IRI in the MRIT2WIHS group were significantly higher than those in the normal group (T2WIHS/normal = 10 (3.1)/4 (0.7), *P* < 0.05), as was axial pain in perioperative local complications (T2WIHS/normal = 5 (1.5)/2 (0.3), *P* < 0.05). After matching, only systemic complications of spinal cord IRI remained significantly more common in the MRIT2WIHS group than in the normal group. There were no significant differences in other perioperative systemic and local complications before and after matching. Furthermore, there were no significant differences in operative time, blood loss, blood transfusion, volume of drainage, antibiotic use, or special treatment of perioperative complications before and after matching.

In the last table, the length of hospital stay in the MRI T2WIHS group was significantly higher than that in the normal group before matching (T2WIHS/normal = (9.3 ± 4.0)/(8.2 ± 3.4), *P* < 0.01) and after matching (T2WIHS/normal = (9.2 ± 3.9)/(8.5 ± 3.7), *P* < 0.01). On the contrary, the improvement of JOA in the MRI T2WIHS group was significantly lower than that in the normal group before matching (T2WIHS/normal = (57.5 ± 38.4)%/(70.7 ± 24.2)%, *P* < 0.001) and after matching (T2WIHS/normal = (58.5 ± 37.8)%/(67.7 ± 23.4)%, *P* < 0.001).

## 4. Discussion

In previous studies, many studies focused on the influence of changes in cervical spinal cord MRI signal on the clinical prognosis of patients, suggesting that high MRIT2WI signal indicates poor cervical spondylotic myelopathy [22, 23]. However, there has been no comparative study on perioperative complications in patients with CSWSCC with the MRI T2WIHS or normal group. In our study, we retrospectively analyzed the clinical data of 913 patients with CSWSCC who were hospitalized for surgery in our hospital over the past 9 years. Randomized controlled trials (RCTS) are considered the gold standard method for eliminating selection bias in comparison studies between groups. To minimize the selection bias of preoperative variables between the two groups, we used propensity matching scoring method and random technique was selected in the matching process. MRI T2WIHS indicated that the spinal cord nerve was severely compressed and edema was obvious and preoperative FG was mostly low (Table 1). In addition, the proportion of males and cervical spine instability were significantly higher compared with the normal group. Finally, the differences of preoperative case characteristics were eliminated after pairing (Table 1).

We have presented that MRI T2WIHS was closely associated with the risk factors of systemic complications during perioperative period. Although there was no significant difference between the two groups, respiratory complications, namely, dyspnea and pneumonia, seemed to be more likely to occur in patients with MRI T2WIHS. A previous large cohort study has shown that preoperative cervical myelopathy is a risk factor for postoperative respiratory complications, and with one case report suggested that cervical myelopathy was the cause of phrenic nerve palsy [24]. Therefore, this indirectly indicates that patients with cervical MRI T2WIHS are more prone to postoperative respiratory complications. As for axial pain, patients with MRI T2WIHS seemed to occur more frequently, although there was no statistical difference after matching. Liu et al. reported that decreased stability of cervical spine structure was an important factor leading to axial pain [25], which was consistent with our study data (Table 1 and Table 2).

As the only complication with significant statistical difference in perioperative systemic complications, the incidence of IRI in patients with MRI T2WIHS was significantly higher than that in patients with normal MRI signal. The surgical treatment of CSWSCC is to relieve the compression of the spinal nerve through surgical decompression. However, due to the local anoxic metabolism changes of the compressed spinal nerve, the sudden increase of blood flow after decompression of the spinal nerve may lead to IRI [26]. According to previous researches, the high signal changes on MRI T2WI indicated swelling and edema of the spinal cord [15, 27]. Additionally, Takahashi et al. reported that MRI T2WIHS may be related to myelomalacia or secondary glial hypertrophy or long-term spinal cord compression [28]. Furthermore, Karadimas et al. claimed that cord decompression was an important factor leading to IRI [17]. Our study suggests that MRI imaging of spinal cord compression changes, such as edema, may exacerbate IRI due to surgical decompression (Figure 1). In addition, further experimental studies are needed to confirm and clarify the mechanism of its occurrence. There were no significant differences in operative time, blood loss, blood transfusion, volume of drainage, antibiotic use, or special treatment of perioperative complications before and after matching.

Regarding hospital stay, the length of hospital stay was more significantly increased in patients with MRI T2WIHS (Table 3). The possible reasons were (1) patients with MRI T2WIHS had relatively obvious symptoms, although there was no significant difference after matching. (2) Our study showed that patients with MRI T2WIHS had a higher incidence of perioperative complications, such as ischemia-reperfusion injury. (3) Data showed that postoperative neurological function improvement was relatively poor in patients with MRI T2WIHS. Previous studies have found that neurological outcomes in patients with MRI T2WIHS are worse than those in patients with normal MRI signal [15, 23]. In our study, it was also confirmed that patients with MRI T2WIHS had poorer perioperative neurological function improvement, which was based on the improvement rate of JOA score (Table 3). Ikegami et al. suggested that spinal cord signal changes (MRI T2WIHS) caused by spinal cord compression could be divided into reversible and irreversible spinal cord injury [23]. Moreover, Vedantam and Rajshekhar pointed out that the longer the spinal cord segment altered by MRI T2 signal, the worse the postoperative prognosis [29].

Our present clinical retrospective study has some shortcomings. First, this study was based on single-center clinical data and is not representative of all patients with CSWSCC who underwent cervical decompression and internal fixation surgery. Second, the data in our study did not reflect the type of MRI signal change (linear or segment, clear or vague) nor the segment length of signal change. Third, the indicators included in the study were not complete enough, such as perioperative VAS (visual analogue scale), NDI (neck disability index), and hospitalization costs. In addition, for MRI T2WIHS, we only recorded imaging features intuitively, without further distinguishing spinal cord edema, spinal cord liquefaction, or other pathological changes leading to it in the spinal cord. Furthermore, the surgeon's own preferences and experience might still influence the results of the study, despite using the propensity matching method.

## 5. Conclusion

Our study confirmed that there was no significant difference in the incidence of perioperative complications in CSWSCC patients with or without MRI T2WIHS, except for the cervical cord IRI. In addition, the JOA improvement rate of patients without MRI T2 signal was significantly better; however, the length of hospital stay was obviously increased in the MRI T2WIHS group. Our research findings will provide good guidance for cervical surgeons to adopt a more scientific and personalized management plan for CSWSCC patients before cervical surgery.

## Figures and Tables

**Figure 1:** An MRI T2WIHS patient (M, 62 y) with CSWSCC presented with postoperative spinal cord IRI. (a–c) Preoperative cervical X-ray, MRI T2WI, and MRI T2 lipid suppression images, respectively, with MRI T2WIHS indicated by the white arrows. (d–f) Postoperative relative images, respectively.

**Table 1:** Features between two groups before and after matching.

	Before propensity score matching			After propensity score matching		
	T2WIHS (*N* = 326)	Normal (*N* = 587)	*P*	T2WIHS (*N* = 312)	Normal (*N* = 312)	*P*
Gender			0.002^∗∗^			0.645
Male	226 (69.3)	256 (43.6)		212 (67.9)	217 (69.6)	
Female	100 (30.7)	331 (56.4)		100 (32.1)	95 (30.4)	
Age			0.126			0.090
60 y	209 (64.1)	416 (70.9)		201 (64.4)	219 (70.2)	
60 y	117 (35.9)	171 (29.1)		111 (35.6)	93 (29.8)	
BMI (kg/m^2^)			0.145			0.252
18.5	25 (7.7)	26 (4.4)		24 (7.7)	16 (5.1)	
18.5~24.9	218 (66.9)	403 (68.7)		207 (66.3)	210 (67.3)	
25.0	83 (25.4)	158 (26.9)		81 (26.0)	86 (27.6)	
Emergency admission			0.459			0.905
Yes	2 (0.6)	5 (0.9)		2 (0.6)	4 (1.3)	
No	324 (99.4)	582 (99.1)		310 (99.4)	308 (98.7)	
Frankel grading			<0.001^∗∗∗^			0.536
C	179 (54.9)	199 (33.9)		165 (52.9)	166 (53.2)	
D	147 (45.1)	388 (66.1)		147 (47.1)	146 (46.8)	
Revision surgery			0.880			0.832
Yes	23 (7.1)	30 (5.1)		19 (6.1)	25 (8.0)	
No	303 (92.9)	557 (94.9)		293 (93.9)	287 (92.0)	
OALL	28 (8.6)	54 (9.2)	0.397	25 (8.0)	30 (9.6)	0.503
OPLL	63 (19.3)	95 (16.2)	0.250	56 (17.9)	51 (16.3)	0.256
Cervical instability	56 (17.2)	56 (9.5)	0.005_∗∗_	42 (13.5)	36 (11.5)	0.260
Diabetes	24 (7.4)	43 (7.3)	0.637	23 (7.4)	26 (8.3)	0.819
Hypertension	68 (20.9)	99 (16.9)	0.202	61 (19.6)	55 (17.6)	0.207
Coronary heart disease	2 (0.6)	6 (1.0)	0.397	2 (0.6)	6 (1.9)	0.145
Liver and kidney dysfunction	1 (0.3)	3 (0.5)	0.603	0 (0.0)	1 (0.3)	0.473
Cerebrovascular disease	6 (1.8)	20 (3.4)	0.270	6 (1.9)	12 (3.8)	0.492
History of malignant tumor	1 (0.3)	4 (0.7)	0.988	1 (0.3)	0 (0.0)	0.855
Osteoporosis	18 (5.5)	37 (6.3)	0.891	16 (5.1)	15 (4.8)	0.609
Ankylosing spondylitis	1 (0.3)	2 (0.3)	0.967	1 (0.3)	1 (0.3)	0.589
Rheumatoid arthritis	3 (0.9)	9 (1.5)	0.265	3 (1.0)	6 (1.9)	0.312
Smoking history	58 (17.8)	80 (13.6)	0.759	55 (17.6)	49 (15.7)	0.387
Other infection	0 (0.0)	5 (0.9)	>0.99	0 (0.0)	4 (1.3)	>0.99
Operative approach			0.958			0.935
Anterior	257 (78.8)	492 (83.8)		249 (79.8)	246 (78.8)	
Posterior	61 (18.7)	84 (14.3)		57 (18.3)	58 (18.6)	
Combined	8 (2.5)	11 (1.9)		6 (1.9)	8 (2.6)	

All data are shown as the mean ± SD and *n* (%) in the table. ^∗^*P* < 0.05, ^∗∗^*P* < 0.01, and ^∗∗∗^*P* < 0.001 displayed in the table. OALL: ossification of anterior longitudinal ligament; OPLL: ossification of posterior longitudinal ligament; BMI: body mass index; T2WIHS: T2-weighted image high signal.

**Table 2:** Systemic and local complications between two groups before and after matching.

	Before propensity score matching			After propensity score matching		
	T2WIHS (*N* = 326)	Normal (*N* = 587)	*P*	T2WIHS (*N* = 312)	Normal (*N* = 312)	*P*
Operating time	97.0 ± 37.4	93.0 ± 33.3	0.901	96.2 ± 36.8	95.8 ± 34	0.495
Bleeding	246.1 ± 425.7	200.0 ± 280.5	0.147	241.7 ± 432.3	199.4 ± 260.3	0.554
Blood transfusion	69.0 ± 356.5	51.6 ± 189.1	0.278	71.1 ± 363.9	48.4 ± 167.6	0.736
Systemic complications						
Dyspnea	4 (1.2)	1 (0.2)	0.076	4 (1.3)	0 (0)	0.341
Pneumoderma	1 (0.3)	0 (0)	>0.99	1 (0.3)	0 (0)	>0.99
Cerebrovascular accident	0 (0)	1 (0.2)	>0.99	0 (0)	1 (0.3)	>0.99
Peptic ulcer	2 (0.6)	5 (0.9)	0.526	2 (0.6)	2 (0.6)	0.380
Dysphagia	5 (1.5)	5 (0.9)	0.878	4 (1.3)	4 (1.3)	0.633
Pneumonia	15 (4.6)	12 (2.0)	0.191	13 (4.2)	4 (1.3)	0.094
Hoarseness	1 (0.3)	3 (0.5)	0.364	1 (0.3)	2 (0.6)	0.380
Sepsis	0 (0)	1 (0.2)	>0.99	0 (0)	0 (0)	0.963
Mental disorder	6 (1.8)	1 (0.2)	0.054	6 (1.9)	0 (0)	0.926
Deep venous thrombosis	1 (0.3)	0 (0)	>0.99	1 (0.3)	0 (0)	0.967
IRI	10 (3.1)	4 (0.7)	0.016^∗^	7 (2.2)	2 (0.6)	0.033^∗^
Sense of girdle	3 (0.9)	0 (0)	>0.99	3 (1.0)	0 (0)	0.943
Local complications						
Axial pain	5 (1.5)	2(0.3)	0.036∗	5(1.6)	2(0.6)	0.179
Palsy of C5	10 (3.1)	12 (2.0)	0.636	9 (2.9)	4 (1.3)	0.931
CSFL	11 (3.4)	14 (2.4)	0.817	9 (2.9)	9 (2.9)	0.887
Esophagostomy	3 (0.9)	1 (0.2)	0.266	2 (0.3)	1 (0.3)	0.669
Incision infection	5 (1.5)	4 (0.7)	0.451	4 (1.3)	4 (1.3)	0.599
Urinary tract infection	0 (0)	1 (0.2)	>0.99	0 (0)	1 (0.3)	>0.99
Local hematoma formation	4 (1.2)	3 (0.5)	0.730	4 (1.3)	1 (0.3)	0.452
Special treatment of complications	4 (1.2)	3 (0.5)	0.891	4 (1.3)	3 (1.0)	0.421
Volume of drainage	166.5 ± 262.1	130.3 ± 167.0	0.494	162.6 ± 260.7	148.6 ± 187.8	0.552
Abnormal antibiotic use	28 (8.6)	37 (6.3)	0.722	24 (7.7)	23 (7.4)	0.915

All data are shown as the mean ± SD and *n* (%) in the table. ^∗^*P* < 0.05, ^∗∗^*P* < 0.01, and ^∗∗∗^*P* < 0.001 displayed in the table. CSFL: cerebrospinal fluid leakage; IRI: ischemia-reperfusion injury; T2WIHS: T2-weighted image high signal.

**Table 3:** Hospital stay and clinical outcomes between two groups before and after matching.

	Before propensity score matching			After propensity score matching		
	T2WIHS (*N* = 326)	Normal (*N* = 587)	*P*	T2WIHS (*N* = 312)	Normal (*N* = 312)	*P*
Hospital stay	9.3 ± 4.0	8.2 ± 3.4	0.001^∗∗^	9.2 ± 3.9	8.5 ± 3.7	0.003^∗∗^
Improvement of JOA	(57.5 ± 38.4)%	(70.7 ± 24.2)%	<0.001^∗∗∗^	(58.5 ± 37.8)%	(67.7 ± 23.4)%	<0.001^∗∗∗^

All data are shown as the mean ± SD and *n* (%) in the table. ^∗^*P* < 0.05, ^∗∗^*P* < 0.01, and ^∗∗∗^*P* < 0.001 displayed in the table. T2WIHS: T2-weighted image high signal; JOA: Japanese Orthopaedic Association. Improvement of JOA = ((postoperative JOA score − preoperative JOA score)/(17 − preoperative JOA score))∗100%.

## Data Availability

The datasets used and/or analyzed during the present study are available from the corresponding authors on reasonable request.

## Abbreviations

CSWSCC: Cervical spondylosis with spinal cord compression
PSM: Propensity score matching
MRI: Magnetic resonance imaging
T2WIHS: T2-weighted image high signal
OALL: Ossification of anterior longitudinal ligament
OPLL: Ossification of posterior longitudinal ligament
CSFL: Cerebrospinal fluid leakage
IRI: Ischemia-reperfusion injury
VAS: Visual analogue scale
NDI: Neck disability index.
